This article has been retracted.

# Clinical Efficacy of Huangkui Capsule plus Methylprednisolone in the Treatment of Nephropathy and the Effect on Urinary Protein and Serum Inflammatory Factors in Patients

**DOI:** 10.1155/2022/6232264

**Published:** 2022-07-06

**Authors:** Weibo Wan, Jingjing Zhou, Rong Lu, Chaoyang Wang, Shuli Hu, Mei Liu, Rong Xiong, Jing Kuang, Xuepeng Fan

**Affiliations:** Department of Critical Care, Wuhan First Hospital of Hubei Province, Wuhan 430000, China

## Abstract

**Objective:**

The study aimed to assess the clinical efficacy of Huangkui capsule plus methylprednisolone in the treatment of nephropathy and the effect on urinary protein and serum inflammatory factors in patients.

**Methods:**

Between June 2017 and July 2020, 90 patients with nephropathy admitted to our hospital were recruited after assessment of eligibility and assigned via the random number table method (1 : 1) to receive either methylprednisolone tablets (observation group) or methylprednisolone tablets plus Huangkui capsules (experimental group). All eligible patients were also given dipyridamole and valsartan. Outcome measures included clinical efficacy, urine protein, hematuria, serum inflammatory factor levels, and adverse reactions.

**Results:**

A higher clinical efficacy was observed in the experimental group versus the observation group (*P* < 0.05). Huangkui capsules resulted in significantly lower levels of urine protein and hematuria in the experimental group versus the observation group after treatment (*P* < 0.05). The serum tumor necrosis factor-*α* (TNF-*α*), interleukin (IL)-6, and monocyte chemoattractant protein-1 (MCP-1) levels in the experimental group were significantly lower than those in the observation group after treatment (*P* < 0.05). Huangkui capsules plus methylprednisolone were associated with a lower incidence of adverse events versus methylprednisolone (*P* < 0.05).

**Conclusion:**

The clinical efficacy of Huangkui capsule plus methylprednisolone in the treatment of patients with nephropathy is remarkable. It can effectively mitigate the inflammatory responses and enhance renal function, with reliable clinical safety, so it is worthy of clinical application.

## 1. Introduction

Chronic kidney disease (CKD) is a common and frequently occurring disease, among which, primary glomerular disease is the most common type of disease leading to CKD in our country. Pathological manifestations include mild glomerular lesions, mesangial proliferative glomerulonephritis, and IgA nephropathy. The occurrence of these diseases is mostly mediated by immune inflammatory response, and local inflammation in the kidney is the central link in the progression of the disease. After the international nephrology community proposed the concept of tertiary prevention and treatment of CKD, the American K/DOQI organization re-established the clinical practice guidelines for CKD in 1999, pointing out that proteinuria is one of the important risk factors for accelerating the progression of CKD [1]. Therefore, effectively controlling proteinuria and protecting renal function are the top priorities in the treatment of CKD.

Drug therapy is the main clinical treatment method for patients with renal disease, and mainstream drugs include angiotensin-converting enzyme inhibitors, angiotensin receptor inhibitors, lipid-lowering drugs, or glucocorticoids [2]. Glucocorticoids and immunosuppressants are mainly used in patients with clinical manifestations of nephrotic syndrome or nephrotic range proteinuria but are not completely suitable for non-nephrotic range proteinuria, and the treatment course of western medicine is long; it is easy to rebound after drug withdrawal. There are also more side effects. Methylprednisolone is an adrenal glucocorticoid that is commonly used in clinical treatment of patients with renal disease [3]. Kidney disease is related to renal damage and the decline of various functional systems, which can further aggravate the disease. Some clinical studies have pointed out that conventional drugs and methylprednisolone tablets have a poor therapeutic effect on patients with renal disease [4] and need to be combined with other drugs to improve the therapeutic effect of patients [5].

Traditional Chinese medicine (TCM) has certain advantages in the treatment of various diseases [6]. In recent years, it has performed well in the treatment of kidney disease patients due to its remarkable curative effect and low side effects [7]. Studies have shown that traditional Chinese medicine has a good effect in improving the clinical symptoms of chronic glomerular disease, controlling proteinuria, protecting renal function, and reducing the side effects of western medicine, especially for patients with proteinuria in the non-nephrotic range. Huangkui capsule is a traditional Chinese medicine with astragalus as the main component, which has the effects of clearing away heat and dampness, detoxification, and swelling [8]. According to “Compendium of Materia Medica” : Huangkui capsule can treat gonorrhea, carbuncle swollen poison, and decoction scald embolism. In addition, due to its sweet and cold medicinal properties, it can also treat burns and scalds [9]. It is also mainly used for various malignant sores and pus that do not heal for a long time. Accordingly, this study recruited 90 patients with nephropathy who were admitted to our hospital from June 2017 to July 2020 and evaluated the clinical efficacy of Huangkui capsules combined with methylprednisolone in the treatment of nephropathy and its effect on urinary protein and serum inflammatory factors.

## 2. Materials and Methods

### 2.1. Baseline Data

Between June 2017 and July 2020, 90 patients with nephropathy admitted to our hospital were recruited after assessment of eligibility and assigned via the random number table method (1 : 1) to an observation group or an experimental group. There were 27 male and 18 female cases in the observation group, aged 22–67 years, with a mean age of (41.27 ± 10.12) years, disease duration of 4–55 months, and a mean disease duration of (22.42 ± 11.62) months. There were 25 male and 20 female cases in the experimental group, aged 23–65 years, with a mean age of (40.96 ± 10.07) years, disease duration of 4–55 months, and a mean disease duration of (22.28 ± 11.39) months. The study/research was approved by the Ethics Committee of the Wuhan First Hospital of Hubei Province, (No.: 2979107).

### 2.2. Inclusion and Exclusion Criteria

The inclusion criteria were as follows: (1) the patients met the diagnostic criteria of clinical nephropathy after Chinese and western medicine diagnoses; (2) the patients were informed and voluntarily cooperated with this study.The exclusion criteria were as follows: (1) patients with other major diseases; (2) patients with psychiatric diseases.

### 2.3. Treatment Methods

The patients in the observation group were orally administered dipyridamole tablets (specification: 30 mg and state drug quantification: H20066585), 3 times/d, 30 mg/d, valsartan capsules (specification: 45 mg and state drug quantification: H20010811) 1 time/d, 90 mg/d, and methylprednisolone tablets (specification: 40 mg and state drug quantification: H2220245) 1 time/d, with an initial dose of 40 mg/day and a maintenance dose of 8 mg/day. The treatment lasted for 10 weeks. The patients in the experimental group were administered Huangkui capsules on top of the treatment in the observation group. The Huangkui capsule (specification: 0.5 g and batch number: Z19990040) was administered 3 times a day, 2 g each time, and the total course of treatment lasts 10 weeks (i.e., 70 days).

### 2.4. Outcome Measures

#### 2.4.1. Clinical Efficacy

Cured: patients' clinical symptoms disappeared, no microscopic hematuria was seen, and the 24 h urine protein amount was less than 0.2 g. Effective: patients' symptoms disappeared, no microscopic hematuria was seen, and the 24 h urine protein amount was more than 0.2 g but decreased by more than 50% compared with before treatment. Ineffective: patients' symptoms did not improve or even worsened.

#### 2.4.2. Urine Protein and Hematuria Level

The detection kits provided by German Desai Diagnostic System Co., Ltd. were used to determine the 24 h urine protein and hematuria level before and after treatment by the colorimetric method of the o-benzene phenol red molybdenum colorimetric method.

#### 2.4.3. Serum Inflammatory Factors

The levels of serum inflammatory factors, including tumor necrosis factor-*α* (TNF-*α*), interleukin-6 (IL-6), and monocyte chemoattractant protein-1 (MCP-1), were determined before and after treatment in the two groups by using the enzyme-linked immunosorbent assay reagents. The experimental kits were purchased from Shanghai R&S Industrial Co.

#### 2.4.4. Adverse Events

Adverse events during treatment including abdominal pain, bloating, dry cough, and dizziness were recorded to calculate the incidence of adverse events. New instances of adverse events/total population were treated during the trial (^*∗*^ 100% = incidence of adverse events).

### 2.5. Statistical Analysis

SPSS 21.0 was used for data analyses, and GraphPad Prism 8 was used for image rendering. The measurement data were expressed as (‾*x* ± *s*) and processed using the *t*-test. The count data were expressed as the number of cases (rate) and analyzed using the chi-square test. Differences were considered statistically significant at *P* < 0.05.

## 3. Results

### 3.1. Baseline Data

Both groups showed the similar baseline data, which were not statistically significant and would not cause too much error in the experimental results (*P* > 0.05). (Table 1).

### 3.2. Clinical Efficacy

The number of effective people in the control group was 35 (accounting for 78% of the total number of the control group), while the number of effective people in the experimental group was 44 (accounting for 98% of the total number of the experimental group), so the clinical effect of the experimental group was better than that of the observation group (*P* < 0.05). (Table 2).

### 3.3. Urine Protein and Hematuria

Huangkui capsules resulted in significantly lower levels of urine protein and hematuria in the experimental group versus the observation group after treatment (*P* < 0.05). (Figure 1).

### 3.4. Inflammatory Factor Levels

The serum levels, TNF-*α*, IL-6, and MCP-1, in the experimental group were significantly lower than those in the observation group after treatment (*P* < 0.05). (Figure 2).

### 3.5. Adverse Events

The number of adverse events in the control group was 10 (22% of the total number of the control group), while the number of people in the experimental group was 2 (4% of the total number of the experimental group), so the probability of adverse events in the experimental group was small, that is, the same as the methyl group. Huangkui capsules plus methylprednisolone had a lower incidence of adverse events compared to prednisolone (*P* < 0.05). (Table 3).

## 4. Discussion

In modern times, the clinical treatment of patients with nephropathy primarily relies on drug therapy, which aims to improve renal function and ameliorate the prognosis [10]. Glucocorticoids can effectively inhibit the inflammatory response of the patient's body to improve the glomerular membrane permeability and the urinary protein level of the patients. Methylprednisolone is a drug commonly used in the clinical treatment of patients with nephropathy and belongs to glucocorticoids [11], which can effectively regulate the cellular and humoral immunity of the patient [12]. The drug also increases the vascular tension of the organism, thus circumventing the capillary overflow situation and relieving the inflammatory response [13]. Clinical studies have shown that patients with kidney disease have structural and functional changes in their kidneys that impair their renal function and that glucocorticoid therapy alone is not sufficient to reduce urinary protein levels and may lead to disease progression. Thus, the monotherapy of methylprednisolone is discouraged in clinical practice [14]. The main ingredient of the Huangkui capsule is Abelmoschus Manihot, which contains active ingredients such as myricetin, quercetin-3 hyperin, quercetin-3-glucoside, and quercetin [15]. Wang et al. confirmed that Huangkui capsules can inhibit glomerular immunity of the organism to abate the inflammatory response, and it also inhibits platelet aggregation to mitigate the impairment of kidney function. In addition, the Huangkui capsule also has the effect of scavenging oxygen free radicals, reducing urine protein, blood urea nitrogen, and muscle libido [16, 17].

The results of the present study showed that Huangkui capsules plus methylprednisolone resulted in significantly better clinical efficacy and lower levels of urine protein and blood urine versus conventional treatment, which indicate that Huangkui capsules plus methylprednisolone feature a remarkable efficacy by effectively enhancing the renal function of the patients. The reason for this can be due to the fact that Abelmoschus Manihot is an anti-inflammatory diuretic, which can effectively reduce the damage to renal tubular and glomerular function in patients [18]. TNF-*α* and IL-6 are common proinflammatory factors, and MCP-1 is a *β*-subgroup chemokine that can produce chemotactic activity on monocytes and induce monocytes and macrophages to secrete lysozyme, thereby aggravating the inflammation of the body [19]. In addition, it can cause fibrotic changes in the kidneys, which can aggravate kidney function damage in the body. The detection of these three inflammatory factors can then effectively reflect the degree of inflammatory damage in the body [20]. The results of the present study showed that patients receiving Huangkui capsules showed significantly lower levels of TNF-*α*, IL-6, and MCP-1, suggesting the effectiveness of Huangkui capsules plus methylprednisolone in improving the inflammatory response in patients with nephropathy [21]. The reason may be that the flavonoids such as myricetin, hyperin, and quercetin in Abelmoschus Manihot exhibit antibacterial and anti-inflammatory functions, improve immunity, and plus clear immune complexes in the circulatory system. Furthermore, Huangkui capsules plus methylprednisolone herein resulted in a significantly lower incidence of adverse events versus methylprednisolone, which may be attributed to the fact that the multiple active ingredients contained in Huangkui capsules constituted the benefits of multitargeted therapy, which complemented the effects of methylprednisolone, thus reducing the occurrence of adverse effects during treatment [22].

To sum up, Huangkui capsules combined with methylprednisolone has a significant clinical effect in the treatment of patients with nephropathy and can effectively reduce inflammation and enhance renal function, which is worthy of clinical application. In addition, the clinical safety of Huangkui capsules combined with methylprednisolone in the treatment of nephropathy has been initially reflected in this experiment, but the number of multicenter, large-sample, randomized clinical trials on this topic is still insufficient. Our next step is to study the dosage interval of different drugs to explore the most effective dose combination, and a more complete treatment system has been established.

## Figures and Tables

**Figure 1:** Comparison of urine protein and hematuria (‾*x* ± *s*). After Huangkui capsule treatment, the levels of urine protein and hematuria in the experimental group were significantly lower than those in the observation group. The symbol^*∗*^ indicates *P* < 0.05.

**Figure 2:** Comparison of inflammatory factor levels (‾*x* ± *s*). The serum levels of TNF-*α*, IL-6, and MCP-1 in the experimental group after treatment were significantly lower than those in the observation group. The symbol^*∗*^ indicates *P* < 0.05.

**Table 1:** Comparison of the baseline data (*n* (%)).

	Observation group (*n* = 45)	Experimental group (*n* = 45)	t or x^2^	*P* value
Gender			0.182	0.67
Male	27	25		
Female	18	20		

Age (years)	22–67	23–65		
Mean age (years)	41.27 ± 10.12	40.96 ± 10.07	0.146	0.884

Disease duration (months)	4–55	5–54		
Mean disease duration (months)	22.42 ± 11.62	22.28 ± 11.39	0.058	0.954

**Table 2:** Comparison of clinical efficacy (*n* (%)).

	Observation group (*n* = 45)	Experimental group (*n* = 45)	x^2^	*P* Value
Cured	21	36		
Effective	14	8		
Ineffective	10	1		
Efficacy (%)	35 (78%)	44 (98%)	9.47	0.002

**Table 3:** Comparison of adverse events (*n* (%)).

	Observation group (*n* = 45)	Experimental group (*n* = 45)	x^2^	*P* value
Abdominal pain	3	0		
Abdominal distension	2	1		
Dry cough	4	1		
Dizziness	1	0		
Total incidence (%)	10 (22%)	2 (4%)	6.154	0.013

## Data Availability

All data generated or analyzed during this study are included in this published article.
